# Screening of Prognostic Markers for Hepatocellular Carcinoma Patients Based on Multichip Combined Analysis

**DOI:** 10.1155/2022/6881600

**Published:** 2022-07-14

**Authors:** Yong Dong, Qian Miao, Da Li

**Affiliations:** ^1^Department of Medical Oncology, Sir Run Run Shaw Hospital, College of Medicine, Zhejiang University, No. 3 Qingchun East Road, Jianggan District, Hangzhou, Zhejiang 310016, China; ^2^Department of Medical Oncology, Quzhou People's Hospital, No. 2, Zhongloudi, Kecheng District, Quzhou, Zhejiang 324000, China

## Abstract

**Methods:**

GSE (14520, 36376, 57957, 76427) datasets were accessed from GEO database. 55 differential mRNAs (DEGs) were obtained by differential analysis based on the datasets. GO and KEGG analysis results indicated that the DEGs were enriched in xenobiotic metabolic process and other pathways. Expression profiles and clinical data of TCGA-LIHC mRNAs were from TCGA database. We established a prognostic model of HCC through univariate and multivariate Cox risk regression analyses. ROC curve analysis was used to examine the prognostic model performance. GSEA analysis was performed between the high- and low-risk score sample groups.

**Results:**

A 4-gene HCC prognostic model was constructed, in which the gene expressions correlated to HCC patients' survival. The AUC value presented 0.734 in the ROC analysis for the prognostic model.

**Conclusion:**

The four-gene model could be introduced as an independent prognostic factors to assess HCC patients' survival status.

## 1. Introduction

Liver cancer is the sixth most commonly diagnosed malignancy, with increasing incidence and mortality year by year [1]. Primary liver cancer consists of 75%-85% hepatocellular carcinoma (HCC) and 10%-15% intrahepatic cholangiocarcinoma along with other rare types [2]. Clinical staging, age, and vascular invasion as important clinical factors may contribute to improvement of survival prediction [3]. Due to the complex molecular mechanism of tumor regulation, traditional clinical information prediction ability is limited. Though a lot of strategies such as hepatectomy, radiofrequency ablation, transcatheter arterial chemoembolization, liver transplantation, and chemotherapy are used in HCC treatment, HCC patient's prognosis is still poor [4]. About 70% of HCC patients have recurrence or metastasis within 5 years after surgery [5]. With the continuous improvement of tumor heterogeneity and molecular mechanism research, new tools like molecular markers are in urgent need for accurate prediction of patient's prognosis.

Genome sequencing technology and data emerged in this genomic era [6]. Microarray and bioinformatics analysis are applied to screen differentially expressed genes (DEGs) at the genomic level, which may aid in the identification of DEGs and pathways correlated with occurrence and development of HCC. Gene chips can rapidly detect DEGs, generate slicing data, and store them in a public database, which is a reliable technology [7]. Great contributions have been made to tumor diagnosis and prognosis prediction. On the basis of these data, valuable evidence can be found for new research. For example, through public databases, more and more potential biomarkers are being mined [8–10]. Feng et al. used lung adenocarcinoma (LUAD) dataset from TCGA and found that LUAD patients expressing high HMGB1 level had dismal overall survival (OS) [11]. Wang et al. take advantage of RNA sequencing (RNA-seq) data from TCGA-KIRC to confirm DEGs [12]. For HCC, Kong et al. selected the top 25% DEGs from the GSE62232 dataset and screened out prognostic-related modules to build protein-protein interaction (PPI) networks, who obtained 5 candidate genes (PCNA, RFC4, PTTG1, H2AFZ, and RRM1) finally [13]. It is indicated that these fresh next-generation sequencing methods and data can screen biomarkers.

Despite the prognostic ability of signature genes being explored by bioinformatics analysis, these prognostic prediction effects are limited due to the heterogeneity of HCC [14]. These prognostic prediction effects are subject to certain challenges, and thus, it is necessary to develop reliable novel signature genes to design a more personalized diagnostic and therapeutic plan. In this study, we downloaded 4 sets of HCC mRNA chip data from GEO database and analyzed them to obtain the differentially expressed mRNAs (DEmRNAs) between HCC tissues and noncancer tissues. Subsequently, biological significance and key pathways of the DEGs were explored through GO and KEGG enrichment analyses. Cox regression analysis, risk assessment, and clinical information analysis helped us find markers that could predict HCC patients' prognoses. Here, a total of 55 DEmRNAs and 4 independent prognostic factors for HCC were identified, which may be candidate biomarkers for HCC, being utilized for prediction of HCC progression and prognosis. A new method for adjuvant therapy of clinical HCC patients was put forward in this study.

## 2. Materials and Methods

### 2.1. Data Downloading and Processing

HCC-related matrix was downloaded from GEO database (https://www.ncbi.nlm.nih.gov/geo/). Criteria for obtaining matrix were (1) human HCC tissue samples, (2) cancer and noncancer samples, (3) the total number of samples ≥ 30, and (4) based on the same sequencing platform. Four groups of HCC mRNA chip data including GSE14520 (normal: 220, tumor: 225), GSE36376 (normal: 193, tumor: 240), GSE57957 (normal: 193, tumor: 240), and GSE76427 (normal: 52, tumor: 115) were selected for this research. The sequencing platform for GSE36376, GSE57957, and GSE76427 was GPL10558 Illumina HumanHT-12 V4.0 chip, and the sequencing platform for GSE14520 was GPL3921 HT_HG-U133A. Then, the combined differential analysis (logFC > |1.0|, padj < 0.05) was done with “limma” (PMID: 25605792) and “RobustRankAggreg” (PMID: 31638362) in R package to identify DEmRNAs in HCC tissues.

The mRNA expression data and clinical data of TCGA-LIHC were downloaded from TCGA database (https://portal.gdc.cancer.gov/). DEmRNA expression and clinical information screened by differential expression analyses were extracted for subsequent validation.

### 2.2. Functional Enrichment Analysis

GO and KEGG enrichment analyses of DEGs were conducted using R package “clusterProfiler” (PMID: 22455463). GO enrichment analysis investigates the biological significance of DEmRNAs, including long-term enrichment analysis of biological processes, molecular functions, and cellular components. KEGG pathway enrichment analysis seeks key pathways closely related to DEmRNAs. *P* value < 0.05 and false discovery rate (FDR) < 0.05 were set as thresholds. *P* value was calculated based on hypergeometric separation.

### 2.3. Cox Regression Analysis and Model Assessment

Univariate and multivariate Cox risk regression analyses were done on DEmRNAs using the R package “survival” [15]. At first, the clinical information provided by TCGA was used to conduct univariate Cox regression analysis on DEmRNAs, and the DEmRNAs with *P* value < 0.01 were selected (omnibus test). Then, these DEmRNAs were further analyzed by multivariate Cox regression analysis to establish a multigene risk model. Samples were divided into high- and low-risk groups by median risk score, and OS of two groups was compared by R package “survival”. To assess the accuracy and predictive value of risk assessment model, we used R package “survivalROC” (PMID: 33790572) to draw receiver operating characteristic (ROC) curves and conduct independent ROC tests for genes in risk assessment model, respectively, to obtain area under curve (AUC) value.

### 2.4. GSEA Analysis for Hub Genes

To investigate pathway changes in the high- and low-risk groups, the GSEA software (V 4.1.0) was utilized to perform KEGG enrichment pathway analysis to explore potential mechanism of action (PMID: 16199517). Normalized enrichment score (NES) and FDR were used to quantify enrichment and statistical significance, respectively [16].

### 2.5. Correlation Analysis of Risk Scores and Clinical Characteristics

The expression levels of feature genes in the high- and low-risk groups were analyzed by using heat map, and their differences in different clinical information and risk score coefficients were analyzed. The performance of risk scores in different tumor stages was analyzed by box plots, and the reliability of the prognostic model in liver cancer was further validated. Kaplan-Meier survival curve was used to assess the effect of the combination of high- or low-risk score and tumor stage on survival rate (log-rank test was introduced for statistical test).

### 2.6. Expressions of Hub Genes and Survival Analysis

GEPIA database (http://gepia.cancer-pku.cn/index.html) is an integration of RNA expression profiles of tumor and normal samples from TCGA and GTEx projects [17], which can be used for individual analysis. Kaplan-Meier plotter is a popular web tool for assessing the impact of a large number of genes on survival based on EGA, TCGA, and GEO databases [18]. In this study, GEPIA was utilized for expression confirmation and survival analysis of hub genes, and log-rank tests were conducted to measure statistical significance.

## 3. Results

### 3.1. Identification of DEmRNAs in HCC

Four datasets GSE14520, GSE36376, GSE57957, and GSE76427 were obtained from GEO database. Subsequently, a differential gene expression analysis was performed among the 4 datasets and then integrated to remove batch effects; finally, 6 significantly upregulated mRNAs and 49 prominently downregulated mRNAs were screened (Figure 1). These DEGs were selected for further analysis.

### 3.2. GO and KEGG Enrichment Analyses for the DEmRNAs

Then, functional enrichment analysis was conducted on above 55 DEmRNAs to explore their potential biological functions. GO enrichment analysis revealed that these genes were mainly concentrated in cellular response to cadmium ion, detoxification of inorganic compound, and cellular response to zinc ion (Figure 2(a)). KEGG unveiled those genes were enriched mainly in mineral absorption, chemical carcinogenesis DNA adducts, and drug metabolism-cytochrome P450 (Figure 2(b)). Therefore, these DEmRNAs may influence the progression of HCC by influencing these biological functions and pathways.

### 3.3. Screening and Verifying the Optimal Prognostic Hub Genes

To screen out hub genes with the best prognosis, we carried out univariate Cox regression analysis on 55 DEmRNAs and selected 20 genes noticeably associated with HCC patients' prognoses (Table 1). Multivariate Cox regression analysis was done on these 20 related genes to establish a risk model of four genes, among which CDC20 was a high-risk factor while CYP2C9, CLEC1B, and LCAT were low-risk factors (Figure 3(a)). Next, patients were assorted into high- and low-risk groups by median risk score. R package “survival” was utilized to compare survival time of two groups, and survival curves were plotted. A significant difference in OS was seen between the two groups, which demonstrated that survival time of patients in the high-risk group was dramatically shorter than the other group, indicating that the risk score could be used for risk grading and prognosis assessment of HCC patients (Figure 3(b)). The ROC curves manifested that AUC value of the model was 0.734 (Figure 3(c)), indicating that the model had a certain accuracy in diagnosing patients' prognoses. Thus, risk scores of these four hub genes were dramatically associated with HCC patients' prognoses.

### 3.4. Functional Analysis of 4 Selected Genes via GSEA

In order to analyze function changes of the high- and low-risk groups, we used the GSEA software to carry out KEGG pathway analysis on the two groups, and the results displayed that compared with the low-risk group, complement and blood coagulation cascade, fatty acid metabolism, peroxidase, and primary bile acid biosynthesis pathways are significantly activated in the high-risk group (Figure 4). These pathways are closely related to the liver and are the major metabolic processes in the liver. Hence, changes in these pathways can affect the metabolic function of the liver. Therefore, we speculated that hub genes may affect the biological function of cancer cells by regulating the metabolic process of the liver, so as to play a role in prognosis.

### 3.5. Relationship between the Hub Genes and Clinical Features

To validate the reliability of the prognostic model, we explored the performance of the risk score on clinical features. Heat map results showed that CDC20 level increased gradually, while CYP2C9, CLEC1B, and LCAT levels decreased gradually, with increased risk score (Figure 5(a)). Significant differences were seen in different grades, pathological stages, and T stages between high- and low-risk group (Figure 5(a)). Survival time of patients with risk score combined with different clinical stages, pathological grades, and T stages was significantly different (Figure 5(b)), which may be reference factors predicting patient's prognosis. With progression of tumor, the risk value increased (Figure 5(c)). This further indicated that the four-gene model could predict the risk of tumors, and the risk scores and some clinical features established by us (stage, grade, T) could be utilized to comprehensively evaluate patient's prognosis.

### 3.6. Analysis of Hub Genes by the Kaplan-Meier Plotter and GEPIA

GEPIA dataset was used to conduct survival and ROC analysis on 4 hub genes in cancer and normal tissues to test significance of the 4 hub genes to patients' prognosis. We searched the Kaplan-Meier OS curves and progression-free survival (PFS) curves of the four genes in the risk model in the GEPIA database and manifested that these four-gene levels had a dramatic impact on OS of patients (Figure 6(a)), among which the HCC patients with high expressions of CLEC1B, CYP2C9, and LCAT presented poor prognosis. Moreover, CDC20, CLEC1B, and LCAT expression levels also had significant effects on PFS (Figure 6(b)). Independent ROC tests were conducted for the four genes in the risk model, and it was noted that the AUC value of each gene reached more than 0.6 (Figure 6(c)). Therefore, the above results suggested that the expressions of these four genes in HCC were related to the progression of cancer and correlated with prognosis, and these four genes could be used as independent prognostic factors for HCC.

## 4. Discussion

Liver cancer is a malignant tumor with different histological characteristics, which is mainly caused by chronic hepatitis virus infection, gene mutation, cell damage, alcoholic liver disease, and aflatoxin poisoning. Despite advances in cancer treatment, prognosis is unfavorable with increasing morbidity and mortality [19]. Most HCC patients without early detection are not suitable for radical treatment, which may be a reason for dismal prognosis. Many studies have demonstrated that biomarkers can determine the progression of cancer. For example, CCND1, c-myc, and RAS mutations, and hypermethylation of CCND2 promoter have been associated with HCC [20, 21]. Splicing changes of NT5E, Sulf1, and SLC39A14 were also associated with HCC [22–24]. All of these factors can be used as markers to predict the progression of HCC. However, the molecular mechanism of HCC is very complex, including many genetic and epigenetic changes, chromosomal aberrations, gene mutations, and alternative molecular pathways [25]. Therefore, potential and efficient diagnostic and therapeutic markers are in great need. Microarray technology enables the exploration of genetic changes in HCC and has been proved to be an effective strategy for mining novel biomarkers in other diseases.

We analyzed four microarray datasets by multichip combined analysis to obtain DEmRNAs between HCC and noncancer tissues. 55 DEmRNAs were identified, containing 6 upregulated genes and 49 downregulated mRNAs. It is well known that main metabolic pathways in the liver include bile acid synthesis, fatty acid metabolism, complement and coagulation cascade, etc., which play a vital role in disease and human homeostasis [26–29]. Therefore, we used GO and KEGG enrichment analyses to explore biological functions and pathway enrichment of DEmRNAs. The results exhibited that DEmRNAs were mainly concentrated in biological functions such as response to exotic biological stimulation, drug catabolism, complement activation, cAMP response, and signaling pathways such as cytochrome P450, drug metabolism, complement and coagulation cascade, fatty acid metabolism, peroxisome, and primary bile acid biosynthesis. Another study has suggested that the activation of complement can promote the tumor [30]. Oxidoreductase activity may lead to antioxidant defense and can encode tumor repressors that are often altered in tumors [31, 32]. The accumulation of bile acids in the liver inhibits cell growth and improves survival [33]. These conclusions are all consistent with our predictions.

Subsequently, Cox regression analysis and the construction of risk model obtained the 4-gene risk model consisting of CDC20, CLEC1B, CYP2C9, and LCAT. The risk values of these four-gene sets were evaluated and verified to be prognostic factors for HCC. We also found from the extensive literature that these hub genes played an essential role in many cancers including HCC. Based on the gene expression and clinical information of liver cancer patients obtained from the TCGA database, Long et al. used univariate, LASSO, and multivariate Cox regression analyses to establish the prognostic model of liver cancer and used GEO database to verify the feasibility of the model. Finally, a prognostic model based on four marker genes is obtained, and the model can predict the overall survival of liver cancer patients [34]. Similarly, in our study, based on 4 GSE datasets in the GEO database, the liver cancer prognostic model was established by univariate and multivariate Cox regression models and finally verified by the GEPIA database. Since we built the model based on multiple gene sets, the results of this study are more reliable to a certain extent as compared with the earlier studies. Dysregulation of cell cycle processes is vital in the development of tumors [20, 35, 36]. CDC20 is an important regulatory factor in the cell cycle process, which forms ubiquitin-proteolytic enzyme complex by binding with APC and participates in the degradation of various proteins to modulate cell cycle process [37]. It has been reported that upregulation of CDC20 may predict the decrease of OS and DFS in HCC patients [38]. Increased CDC20 in HCC was related to gender, differentiation, and TNM stage [39], which is similar to our results. Through risk model, we manifested that CDC20 was a high-risk factor and was also associated with clinical features. CYP2C9 is a drug metabolism enzyme and is a decreased low-risk factor in HCC [40]. Shuaichen and Guangyi have discovered that CYP2C9 may promote the development of HCC, especially can be a diagnostic biomarker in drug metabolism [41]. CLEC2 is expressed in platelets and some hematopoietic cells. Wang et al. have put forward that CLEC2 inhibits gastric cancer metastasis, prevents the activation of AKT and glycogen synthase signals, and affects the invasion and expression of EMT markers, which can be a potential biomarker in gastric cancer [42]. However, fewer studies on CLEC2 in HCC have been reported. So, our study provided a data source for the role of this gene in HCC. Finally, LCAT is the only enzyme that can esterify cholesterol in plasma, which determines maturation of high-density lipoprotein as a key enzyme for reverse cholesterol transport with reports of its role in atherosclerosis, cholesterol deposition, and kidney [43–45]. Besides, Russell et al. have pointed out that LCAT plays a role as a diagnostic marker in epithelial ovarian cancer [46]. It can also predict OS of HCC [47]. In conclusion, the four hub genes found in this study played a crucial role in HCC. These genes also function in pathways such as complement and blood coagulation cascade, fatty acid metabolism, peroxisome, and primary bile acid biosynthesis. Their expressions in HCC will indirectly affect the changes of these pathways, thus affecting the incidence of HCC, which fully illustrates the importance of these hub genes of HCC progression.

Taken together, we attempted to screen DEmRNAs that may be related to HCC occurrence and development. 55 DEmRNAs and 4 hub genes had been identified as diagnostic biomarkers for HCC, which offered an effective basis for the treatment of HCC. But this experiment still has certain limitations. This study only conducted a pure bioinformatics analysis through the GEO database, further verification in multicenter clinical trials, and prospective studies is required. Nevertheless, biological functions of these genes in HCC need further study.

## Figures and Tables

**Figure 1:** Heat map of DEGs screened by combined analysis of 4 datasets from GEP database. The numbers in the grids represent the fold changes of genes in different datasets between the tumor group and the normal group.

**Figure 2:** GO and KEGG pathway analyses of DEmRNAs in HCC: (a, b) GO and KEGG enrichment analyses of DEGs.

**Figure 3:** Constructing and verification the prognostic model. (a) Forest map of the 4-gene prognostic model established by multivariate Cox risk regression analysis; (b) Kaplan-Meier OS curves for the high- and low-risk groups are plotted based on risk score. Horizontal axis: survival time; vertical axis: overall rate; red line: high-risk samples; blue line: low-risk samples. (c) ROC curves based on the risk model.

**Figure 4:** GSEA pathway enrichment results based on median risk score grouping.

**Figure 5:** Analysis of DEmRNAs and clinical relationship and patients' prognosis. (a) Heat map of 4 gene expressions in the high- and low-risk groups of risk model and clinicopathological differences between the two groups; (b) OS curves combined risk score and the patients' different tumor stages, with the horizontal axis representing survival time and the vertical axis representing OS rate. Different color curves represent different combinations of risk and tumor stage. (c) Boxplots of differences in risk scores of different clinical stages, grades, and T stages.

**Figure 6:** Analysis of hub genes by the Kaplan-Meier plotter and GEPIA. (a, b) Kaplan-Meier OS curves and PFS curves of four genes in the risk model are retrieved in the GEPIA database. Horizontal axis: survival time; vertical axis: survival rate; red line: high-expression group; blue line: low-expression group. (c) Independent ROC curves of four genes in the risk model for HCC patient's prognosis.

**Table 1:** Univariate Cox regression analysis screened genes that were significantly associated with the prognosis of HCC patients.

Gene	HR	*z*	*P* value
CDC20	1.303474527	4.659540595	3.17*E*-06
LCAT	0.800676874	-4.422698682	9.75*E*-06
DNASE1L3	0.834137148	-4.228589383	2.35*E*-05
GHR	0.813122352	-4.187942095	2.81*E*-05
CYP2C9	0.887041102	-4.126833672	3.68*E*-05
ANXA10	0.877021937	-3.969016876	7.22*E*-05
SPP2	0.907350691	-3.964707036	7.35*E*-05
SLC10A1	0.914033265	-3.67849838	0.000234611
SLC22A1	0.909870575	-3.598475946	0.000320087
AFM	0.902676346	-3.557458905	0.00037446
TAT	0.912717953	-3.472545816	0.000515547
ADH1B	0.901724063	-3.429051233	0.000605695
KLKB1	0.842899464	-3.320604451	0.000898227
VIPR1	0.851232022	-3.312650071	0.000924165
TOP2A	1.210739633	3.308652423	0.000937461
RDH16	0.903679968	-3.278095563	0.0010451
CLEC1B	0.860469147	-3.090652798	0.00199717
FCN3	0.8707386	-2.958448406	0.00309192
C7	0.919120279	-2.896960425	0.003767973
IGFALS	0.912348703	-2.779238461	0.005448651

## Data Availability

The data used to support the findings of this study are available from the corresponding author upon request.
